# The Association between Physical Exercise during Pregnancy and Maternal and Neonatal Health Outcomes: A Systematic Review and Meta-Analysis of Randomized Controlled Trials

**DOI:** 10.1155/2022/3462392

**Published:** 2022-08-21

**Authors:** Yangling Wang, Liangjiao Wu, Xiaomei Wu, Changna Zhou

**Affiliations:** ^1^Department of Obstetrics, The First Affiliated Hospital of Hainan Medical University, Haikou 570102, China; ^2^Department of Gynaecology and Obstetrics, Chengmai County People's Hospital, Chengmai, 571900, China; ^3^Department of Gynaecology and Obstetrics, Dongfang People's Hospital, Dongfang 572600, China

## Abstract

**Objective:**

To explore the effect of exercise during pregnancy on the maternal and neonatal health outcomes.

**Methods:**

Eligible papers were systematically retrieved from PubMed, Embase, OVID, and ScienceDirect. Two researchers independently extracted the primary endpoints from the included literature. Random-effect model or fixed-effect model were utilized to generate and compute relative risk and mean difference, as appropriate. Publication bias was quantified and assessed using the funnel plot with Egger's test.

**Results:**

This study included 13 literatures with a total of 3047 pregnant women with gestational weeks more than 10 weeks. The incidence of vaginal delivery was significantly higher in the intervention group than that in the control group (28.7% vs 23.3%, *P* < 0.001). The differences of duration of the first stage and second stage of labor between the interventional group and control group were both statistically insignificant (mean difference: 27.92, 95% CI: − 70.60, 14.7, *P* = 0.20; mean difference: 0.63, 95% CI: − 4.47, 5.74, *P* = 0.81). In addition, there were no significant differences with regard to gestational age at delivery (mean difference = −0.23, 95% CI: − 1.29, 0.83, *P* = 0.67), Apgar score (mean difference = 0.06, 95% CI: − 0.13, 0.26, *P* = 0.53), and birth weight (mean difference = −23.78, 95% CI: − 60.66, 13.11, *P* = 0.21) between the 2 groups. Women in the intervention group were more likely to experience vaginal delivery than the control group (RR = 1.27, 95% CI: 1.04, 1.55, *P* = 0.01).

**Conclusions:**

Physical exercise during pregnancy could improve the incidence of natural labor.

## 1. Introduction

Regular aerobic exercise is essential for maintaining healthy. Exercise during pregnancy is also vital because women of childbearing age have a significantly higher risk of developing gestational diabetes that is highly related to weight gain and altered hormone metabolism during pregnancy. The American College of Obstetricians and Gynecologists recommended 30 minutes of moderate-intensity aerobic exercise every day for pregnant women without obstetric or other complications in 2002 [1]. In fact, many studies have shown that exercise during pregnancy can significantly reduce the risk of placenta previa [2], gestational diabetes [3], preterm delivery [4], and postpartum depression [5]. Exercise can effectively improve the tolerance of labor pain during delivery and postpartum physical function and prevent weight gain during pregnancy. On the contrary, a host of studies have also reported that exercise intervention during pregnancy also impacts the duration of labor, which is highly correlated with the health outcomes of pregnant women and newborns [6]. If the duration of the first stage of labor is prolonged, the fetal head may be squeezed by the birth canal, resulting in a decrease in Apgar score and even stillbirth [7]. The prolonged duration of the second stage of labor may increase the risk of obstetric canal laceration, cesarean section, and pelvic floor muscle injury. Therefore, it is of great clinical significance to determine health interventions that reduce the time of labor and improve the health outcomes of mothers and infants.

Although regular exercise can improve physical health, the effect of exercise during pregnancy on the maternal and neonatal outcome remains controversial [8, 9]. For example, Perales et al. found that the exercise during pregnancy did not increase the incidence of vaginal delivery [10], while other studies have come to the opposite conclusion [11–13]. Therefore, in view of the increasing number of randomized controlled trials (RCT) in recent years to explore the impact of exercise during pregnancy on maternal and neonatal health outcomes [12, 14, 15], we aimed to quantify the effect of exercise intervention during pregnancy on the health outcomes of newborns and pregnant women through systematic review and meta-analysis, thus providing clinical evidence for preventing adverse health outcomes in pregnant women and newborns.

## 2. Methods

### 2.1. Literature Search

The databases of PubMed, EMBASE, ScienceDirect, and OVID were used for literature retrieval from inception to May 15, 2022. The search keywords were (“exercise” OR “aerobic” OR “physical activity”) AND (“Pregnancy”[Mesh Terms OR “Pregnant”) AND (“maternal outcome” OR “neonate outcome” OR “Apgar” OR “delivery∗” OR “labor” OR “gestational age”).

### 2.2. Literature Screening

Retrieved literatures were subject to the following inclusion and exclusion criteria. Inclusion criteria are as follows: (1) The study design was a RCT. (2) The study population was adult pregnant women with gestational weeks longer than 10 weeks. (3) The intervention method studied was regular exercise, including aerobic exercise, resistance exercise, yoga, and swimming. The control group received no exercises. (4) The primary endpoint of the study included at least one of the following six categories: duration of the first stage of labor, duration of the second stage of labor, mode of delivery, gestational age at birth, birth weight and newborn Apgar score.

Literature exclusion criteria are as follows: (1) Studies with no clear definition of intervention, short follow-up time, or the control group also received exercise. (2) Studies with population overlap. (3) The sample size of the interventional group or the control group was less than 20. (4) Non-original articles, such as comments, academic conferences, reviews, case reports. (5) Studies with Newcastle-Ottawa Scale (NOS) score less than 5. This study did not limit the characteristics of pregnant women, such as age, body mass index, prior history of diabetes, hypertension, or other chronic diseases, and whether they are primiparas.

### 2.3. Document Data Sorting and Evaluation

YL. W and LJ. W independently extracted the following data from the included literature: study type, number of patients, primary endpoint indicators such as the duration of the first stage of labor and the duration of the second stage of labor, mode of delivery, gestational age at birth, birth weight, and neonatal Apgar score. The continuous variable and binary variable were expressed as mean difference ± standard deviation and ratio of the number of events in the intervention group and the control group, respectively, as shown in Table 1. The NOS was applied to evaluate the methodological quality of all the included literature. Those with a score below 5 were considered at high-risk for bias, whereas those with a score above 8 were considered at low-risk for bias. When discrepancies emerged between the 2 investigators emerged, an agreement could be reached through discussion with the third researcher.

### 2.4. Statistical Methods

Data analysis and merging in this study were done using STATA 17.0 software, and Endnote X9 was used for literature management. The Cochran's Q and *I*^2^ statistics were used to assess the magnitude of heterogeneity between studies. For *I*^2^ > 50%, the random-effect model based on restricted maximum likelihood method was used; otherwise, the fixed-effect model based on the inverse variance model was used. In addition, the funnel plot was applied to measure publication bias in the meta-analysis. The geometric symmetry of the funnel plot was assessed using Egger's and Begg's tests. All hypothesis tests were considered statistically significant at *P* < 0.05, and all hypothesis tests were two-sided.

## 3. Results

### 3.1. Search Results and Literature Characteristics

A total of 360 relevant literatures were retrieved. According to the inclusion and exclusion criteria, 13 studies with 3047 pregnant women were finally included in the meta-analysis. Detailed process of literature retrieval and screening was presented in Figure 1. Among the 13 studies, 9 reported the duration of the first stage of labor, 8 reported the duration of the second stage of labor, 4 reported the indicators of gestational age at birth, 8 evaluated the Apgar score 5 minutes after birth, and 10 recorded the newborn birth weight and the mode of delivery. According to the Cochrane systematic evaluation system, 2 studies did not describe the grouping concealment and blind method of randomized grouping, which was considered to have a moderate risk of bias, and the rest of the literature had a minimal risk of bias. The NOS score ranged from 5 to 8, including 8 low-risk bias literature, 3 medium-risk bias literature and 2 high-risk bias literature.

### 3.2. Duration of the First Stage of Labor

A total of 2199 children in 9 studies were pooled for the duration of the first stage of labor. The random effect model was used to combine the mean difference, given the high degree of heterogeneity (*H*^2^ = 7.57, *I*^2^ = 86.79%, *P* = 0.20). The results of the meta-analysis (Figure 2) showed that compared with the control group, the duration of the first stage of labor of pregnant women with exercise intervention during pregnancy was statistically insignificant (mean difference: − 27.92, 95% CI: − 70.60, 14.76, *P* = 0.20). The funnel chart (Figure 3) showed no obvious publication bias.

### 3.3. Duration of the Second Stage of Labor

A total of 8 studies with 2119 pregnant women were included in this study. The random effect model was used to combine the mean difference in the presence of high heterogeneity (*H*^2^ = 5.88, *I*^2^ = 83.00%, and *P* = 0.81). The meta-analysis results (Figure 4) showed that the duration of the second stage of labor did not differ significantly between the interventional and control group (mean difference: 0.63, 95% CI: − 4.47, 5.74, *P* = 0.81). No obvious publication bias was observed (Figure 5).

### 3.4. Gestational Age at Birth

A total of 1383 patients in 4 publications were included in this study. The fixed-effect model was applied to combine mean difference in the presence of low degree of heterogeneity (*H*^2^ = 1.11, *I*^2^ = 10.10%, and *P* = 0.67). The meta-analysis (Figure 6) found no significant differences with regard to the gestational age at birth between the interventional group and the control group (mean difference = −0.23, 95% CI: − 1.29, 0.83, *P* = 0.67). There was no obvious publication bias (Figure 7).

### 3.5. Mode of Delivery

Meta-analysis (Figure 8) using the random-effect model (*H*^2^ = 5.74, *I*^2^ = 82.56, *P* = 0.01) suggested that compared with the control group, pregnant women with exercise intervention were significantly more likely to have spontaneous labor (RR = 1.27, 95% CI: 1.04, 1.55, *P* = 0.01). No obvious publication bias was noted (Figure 9).

### 3.6. Apgar Score

A total of 2373 newborns in 10 studies were included in this study. The results of the meta-analysis (Figure 10) with the random-effect model (*H*^2^ = 8.84, *I*^2^ = 88.69%, and *P* = 0.53) showed the newborn Apgar score between the interventional and control group was statistically insignificant (mean difference = 0.06, 95% CI: − 0.13, 0.26, *P* = 0.53). The funnel chart (Figure 11) demonstrated no obvious publication bias.

### 3.7. Birth Weight

The heterogeneity test results of the 10 publications with 1363 participants were *H*^2^ = 1.00, *I*^2^ = 0.00%, and *P* = 0.21. The fixed-effect model was then used. There was no significant differences with regard to the birth weight between the 2 groups (mean difference = −23.78, 95% CI: − 60.66, 13.11, and *P* = 0.21, Figure 12). There was no publication bias (Figure 13).

## 4. Discussion

This study showed that exercise intervention during pregnancy would increase the incidence of natural delivery and newborn Apgar score. The time of the first stage of labor and newborn birth weight in the exercise intervention group was shortened by about 28 minutes and 23.78 g, respectively, despite these differences were statistically insignificant. Hopkins and Cutfield [23] found that the most far-reaching impact of exercise during pregnancy on the health status of newborns may be derived from the reduction of birth weight. In addition, some studies have shown that moderate birth weight reduction is positively related to a decrease in the risk of childhood obesity [24–26]. Compatibly, the newborns in the intervention group had lower birth weight and higher Apgar scores in the present study. Although prior studies suggested that low birth weight is also related to a series of health risks, the main reason against pregnant women from exercising properly during pregnancy is that exercise leads to the diversion of maternal oxygen and nutrients to skeletal muscle rather than to the fetus, which may affect the normal development of the fetus [27]. Nonetheless, the study by Sanabria-Martínez et al. [28] showed that the reduction of neonatal birth weight caused by exercise intervention during pregnancy was within the normal range and had no additional health hazard to the newborn. Some scholars believe that exercise during pregnancy may increase the risk of preterm birth, which is a leading cause of neonatal mortality [29], by increasing the level of norepinephrine. Norepinephrine has been shown to stimulate the uterine myometrium and induces preterm birth [30]. Increased risk of preterm birth has been demonstrated in a prior meta-analysis by Kramer and McDonald [31]. However, it is limited by small sample size that included three RCTs, which might lead to insufficient statistical power. Our study showed that exercise intervention during pregnancy did not affect the gestational weeks of newborns at birth, which was consistent with the conclusion of the 2012 meta-analysis [32] and the 2015 Cochrane meta-analysis [33].

According to the exercise guidelines of the American women's and children's Association [34], Poudevigne et al. recommended that reduced exercise intensity for pregnant women Resistance training can enhance pelvic floor muscles and improve pelvic stability, thus making pelvic floor muscles easier to relax during delivery and improving the position of the fetus in the birth canal. A host of factors affect the duration of delivery, such as the number of births and the time of the initiation of exercise intervention. The duration of the first stage of labor of the primipara was significantly longer than that of the multipara. The study by Zarezadeh et al. only included the primipara [18]. Therefore, it remains unclear at which stage of pregnancy does exercise intervention has the most significant impact on the health outcomes of the mother and fetus. In addition, some studies have suggested that pregnant women who have habits of regular exercise also have significantly higher exercise volume than women who have less exercise frequency in the early stages of pregnancy [35]. Therefore, studies would be more extrapolative by dividing study population into subgroups according to exercise habits, primipara/multipara, and the time of the exercise intervention.

This study suffers from several limitations: (1) The sample size of some RCTs included in this study was small. Only three studies had a sample size of more than 100 cases [12, 15, 17]. (2) Some included studies did not clearly and completely clarify the specific methods of blinding and randomization. (3) Significant heterogeneity in the definition of exercise intervention, such as frequency, intensity, duration of exercise, and the gestational week for exercise intervention, were noted. (4) In some studies, the study population was limited to primiparas, while in others, the study population also included multiparas. Therefore, we cannot definitively exclude the effect of this possible confounding factor. (5) There were also differences in terms of whether the intervention was carried out under the researcher's supervision. Some studies used self-report results to evaluate the intervention, while exercise intervention in others was performed under the researcher's supervision. Therefore, the former might underestimate or overestimate the duration and intensity of exercise during pregnancy, thus introducing potential bias. (6) Differences in the distribution of other factors affecting the birth weight of newborns, such as exposure to environmental factors during pregnancy (noise, air pollutants, smoking, and mental health status of pregnant women during pregnancy) between the interventional and the control group were not reported in most studies.

In conclusion, our study results suggested that exercise intervention during pregnancy increased the incidence of natural delivery and was not associated with increased the health risks or adverse birth outcomes for perinatal pregnant women.

## Figures and Tables

**Figure 1:** Prism flow chart. Process of meta-analysis for screening included literatures.

**Figure 2:** Forest map of the effect of exercise intervention during pregnancy on the duration of the first stage of labor.

**Figure 3:** Funnel chart of the effect of exercise intervention during pregnancy on the duration of the first stage of labor.

**Figure 4:** Forest map of the effect of exercise intervention during pregnancy on the duration of the second stage of labor.

**Figure 5:** Funnel chart of the effect of exercise intervention during pregnancy on the duration of the second stage of labor.

**Figure 6:** Forest map of the effect of exercise intervention during pregnancy on gestational age at birth.

**Figure 7:** Funnel chart of the effect of exercise intervention during pregnancy on gestational age at birth.

**Figure 8:** Forest map of the impact of exercise intervention during pregnancy on labour mode.

**Figure 9:** Funnel chart of the impact of exercise intervention during pregnancy on labour mode.

**Figure 10:** Forest map of the effect of exercise intervention during pregnancy on Apgar score.

**Figure 11:** Funnel chart of the effect of exercise intervention during pregnancy on Apgar score.

**Figure 12:** Forest map of the effect of exercise intervention during pregnancy on birth weight.

**Figure 13:** Funnel chart of the effect of exercise intervention during pregnancy on birth weight.

**Table 1:** Basic characteristics of the literature included in the analysis.

Authors	Study type	Sample size		Duration of the first stage of labor		Duration of the second stage of labor		Gestational age at birth		Spontaneous labor		Apgar score		Birth weight		NOS
		Intervention group	Control group	Intervention group	Control group	Intervention group	Control group	Intervention group	Control group	Intervention group	Control group	Intervention group	Control group	Intervention group	Control group	
Salvesen et al. (2014) [16]	RCT	31	31	373 ± 266	377 ± 373	44 ± 27	38 ± 24	NA	NA	NA	NA	NA	NA	NA	NA	7
da Silva et al. (2017) [17]	RCT	204	407	NA	NA	NA	NA	NA	NA	NA	NA	NA	NA	3244 ± 424	3254 ± 457	6
Sanda et al. (2018) [12]	RCT	295	294	293.4 ± 201	257.1 ± 181	40.5 ± 25	41.5 ± 24.1	279 ± 12	279 ± 13	NA	NA	9.6 ± 0.7	9.4 ± 1.1	3410 ± 486	3449 ± 539	7
Zarezadeh et al. (2016) [18]	RCT	40	40	329.86 ± 220.68	451.3 ± 187.99	NA	NA	NA	NA	34	14	NA	NA	NA	NA	6
Toosi et al. (2016) [11]	RCT	60	60	252 ± 84	288 ± 54	48.9 ± 11.9	51.6 ± 10	274 ± 8	276 ± 6	41	29	9.3 ± 1.3	10 ± 1.6	3185 ± 453	3175 ± 392	8
Ghodsi et al. (2014) [19]	RCT	40	40	299.6 ± 126.87	147.8 ± 40	29.5 ± 13.99	32.5 ± 13.68	NA	NA	35	35	NA	NA	3059 ± 339	3255 ± 456	8
Price et al. (2012) [20]	RCT	31	31	555 ± 300	504 ± 204	47.4 ± 36	28.4 ± 12.5	NA	NA	27	19	9 ± 0.5	8.7 ± 0.5	3329 ± 519	3308 ± 103	8
Rodriguez et al. (2017) [21]	RCT	50	50	NA	NA	NA	NA	NA	NA	45	23	NA	NA	3361 ± 361	3417 ± 473	8
Ghandali et al. (2021) [14]	RCT	55	55	110 ± 70.94	164 ± 99.81	33.4 ± 24.51	50.36 ± 38.59	NA	NA	45	42	9.94 ± 0.24	9.88 ± 0.38	NA	NA	7
Garnaes et al. (2017) [13]	RCT	38	36	NA	NA	NA	NA	NA	NA	29	29	9.6 ± 0.5	9.4 ± 1.2	3719 ± 695	3912 ± 413	***7***
Murtezani et al. (2014) [22]	RCT	30	33	NA	NA	NA	NA	NA	NA	22	17	8.7 ± 0.8	8.2 ± 0.5	3250.8 ± 465.0	3237.9 ± 368.9	7
Barakat et al. (2018) [15]	RCT	255	253	462.83 ± 208.37	409.15 ± 185.74	36.21 ± 25.93	33.23 ± 22.53	278.5 ± 11	277.79 ± 8.57	139	115	9.8 ± 0.5	9.94 ± 0.85	3273 ± 415	3256 ± 466	8
Perales et al. (2016) [10]	RCT	83	83	399 ± 322.1	537.4 ± 409.3	40.6 ± 42.8	37.4 ± 44.7	277 + 8.8	277.9 ± 8.3	69	71	9.8 ± 0.5	9.9 ± 0.2	3183 ± 446	3232 ± 383	8

## Data Availability

The data used to support the findings of this study are available from the corresponding author upon request.
